The article "Performance Index Based on Predicted Auditory Reaction Time Analysis for the Evaluation of Human-Machine Interface in Flight Control" was published in 2022. Journal: Comput Math Methods Med.

# Performance Index Based on Predicted Auditory Reaction Time Analysis for the Evaluation of Human-Machine Interface in Flight Control

**DOI:** 10.1155/2022/4661156

**Published:** 2022-04-12

**Authors:** Weiwei Yu, Dian Jin, Xinliang Yang, Feng Zhao, Haiyang Wang, Ran Peng

**Affiliations:** ^1^School of Mechanical Engineering, Northwestern Polytechnical University, Xi'an, 710072, China; ^2^Avionics Research Institute, Chinese Flight Test Establishment, Xi'an, 710089, China

## Abstract

With the rapid development of complex equipment, such as airplanes, the appropriate design of the human-machine interface is often upgraded, thus emerged many methods to evaluate whether such an upgrade is effective. Most researches focus on the time accumulation effect of the human state during the interaction to evaluate the interface. However, in the aviation application, the performance of the pilot's instantaneous reactions also reveals the design efficiency of the interface, since the difficulty level of obtaining the useful information would severely influence the reaction time in some voice command tasks or emergency situations. Besides, there are so many flight scenarios that are impossible to be simulated in experiments or in a laboratory environment. Also, voice commands are too numerous to be traversed simulated. This paper introduced predicted auditory reaction time as an index to evaluate human-machine interface design. The proposed method has two advantages. On the one hand, it effectively measures the pilot's auditory reaction time based on the eye movement tracking; thus, the data can be taken in flight task scenarios, and the experiment would not cause interference to the subjects. On the other hand, a prediction model is proposed, in which the pilot's reaction time under more generalized voice command can be estimated based on a small-size sample set.

## 1. Introduction

Human-machine (computer) systems refer to the system composed of humans and machines and fulfill some functions through the interaction between humans and machines [1]. With the rapid development of complex equipment, such as airplanes and remotely piloted aircraft (RPA), the appropriate design of the human-machine interface plays a crucial role in harnessing the powerful capabilities of equipment [2]. In common cases, the interface of upgraded equipment is designed or modified based on the original interface of the previous generation, while adding new functions. However, the simple interface modification or updates will not give full play to the capabilities of a new generation of equipment. Sometimes, the interface design may cause user failures to obtain critical information [3] or give rise to malfunctions of cognition and decision-making among operators, which may lead to accidents [4]. Thus, many methods called usability evaluation emerged, aimed at evaluating whether such an upgraded human-machine interface is effective.

The article "Performance Index Based on Predicted Auditory Reaction Time Analysis for the Evaluation of Human-Machine Interface in Flight Control" was published in 2022. Journal: Comput Math Methods Med.

There are methods based on analyzing the static attributes of the interface. In [5], the color and luminance contrast in information coding was discussed in Air Traffic Control (ATC) display systems. A prototype color palette that used color coding to prioritize display information while maintaining good legibility was presented. The Human Algorithm Knowledge-based layout Design method (HAKD) was proposed to deal with the problem of layout design [6]. HAKD took the evolutionary algorithm (e.g., genetic algorithm) as the algorithm foundation, in which human-provided artificial layout schemes (artificial solutions) and layout diagrams afford prior knowledge solutions, and the evolution algorithm produced novel algorithm solutions. Thus, human intelligence, computer intelligence (evolution algorithm), and prior knowledge extracted from layout diagrams were fused for problem-solving.

However, the researches above paid more attention to the static attributes of the interface, and the dynamic factors of humans were seldom taken into consideration. Thus, researches based on the experiment which regarded human performance, either from the aspect of work performance evaluation or the mental workload evaluation, were adopted.

In performance evaluation, a cognitive walkthrough is one method. The developers of an interface walked through the interface in the context of core tasks that a typical user would accomplish. The actions and feedback of the interface were compared to the user's goals and knowledge, and discrepancies between the user's expectations and the steps required by the interface were noted [7]. With the development of technology, eye-tracking became one of the most precise and objective methods of usability studies [8] and was believed to be an efficient method to evaluate the design of the human-machine interface [9]. It was discovered that well-organized functional grouping resulted in shorter scan paths, covering smaller areas. An evaluation method called DEMIS was demonstrated [10]. Two effectiveness measures included the fixation-to-importance ratio (FIR) which represented attentional resources spent on an information source compared to the importance of the information source, and selective attention effectiveness (SAE) which incorporated FIRs for all information sources was proposed. Then, difficulties caused by a poor HMI design were evaluated by a focused interview based on the FIR evaluation.

The article "Performance Index Based on Predicted Auditory Reaction Time Analysis for the Evaluation of Human-Machine Interface in Flight Control" was published in 2022. Journal: Comput Math Methods Med.

Several researches are grounded on measuring the mental workload (MWL) of users to evaluate the user interface design. In engineering application, the NASA Task Load Index (TLX) was adopted as one of the indexes measuring the MWL [11]. It collected subjective workload scores based on a weighted average rating of six factors, which included mental demand, physical demand, temporal demand, own performance, effort, and frustration level. The results showed that the design style of the human-machine interface affected different factors of the operator's workload. Another multi-index evaluation method developed on performance measures, subjective rating, and physiological measure was used to evaluate MWL of operators [12]. It pointed out that interface design had a significant effect on operators' MWL in nuclear power plants. Same in the domain of nuclear power plant interface design, fuzzy comprehensive evaluation theory was adopted in [13] for assessment of interface designs. This method was validated in achieving the quick and accurate assessment of different display interfaces when considering the operators' MWL. In the domain of Air Traffic Control (ATC), [14] used operator's behavior and EGG/ERP to measure the cognitive load and also achieved the effective evaluation of the interface design.

Most of the previous methods based on operation performance or mental workload evaluation considered the time accumulation effect of the human state during the interaction. However, the performance of human instantaneous reactions also reveals the design efficiency of the interface, since the difficulty level of obtaining the useful information would severely influence the response time in some voice commands or emergency tasks. For example, in the application of the flight control interface, for some tasks, especially high maneuverability mission, after voice receiving commands, it is critical for pilots to understand the commands and perform quickly in highly dynamic flight scenarios. The reaction speed may affect the task performance of the whole mission [15]. Also, in the case of special situation handling during the flight, after receiving the auditory warning/alarming signal, the pilot has to obtain useful information from the interface as quickly as possible to avoid the accident [15]. Therefore, in the above application scenario, it is very necessary to propose the reaction time (RT) as one of the indexes to evaluate the user interface.

The pilot's RT is related to his proficiency; for example, expert pilots show less RT [16]. But for the same expert pilot, his RT for certain voice commands can reveal the accessibility of the useful information that the interaction interface provides to the user [17]. RT is commonly defined as the time interval between a stimulus and a reaction, which can be used as an index to evaluate the human-machine interface. In [18], RTs together with mental workload and subjective feedback were used to evaluate the agricultural machine user-centered interface. Significant differences were found in RT between two user interfaces, which showed that RT can be an index to measure the usability of an interface. Considering that the interaction interface may impact the user's efficiency of obtaining useful information, the user's response time for answering the questions related to the information presented on an interface was adopted to infer the situation awareness attained by the user. Higher response time was associated with lower situation awareness. Besides the study on auditory RT, the RT of visual warning, auditory warning, tactile warning, and any combination of these three types of signals were regarded as the indexes to assess the user's interface [19].

The article "Performance Index Based on Predicted Auditory Reaction Time Analysis for the Evaluation of Human-Machine Interface in Flight Control" was published in 2022. Journal: Comput Math Methods Med.

Although these studies have certain practical significance and provide good guidance to evaluate the design of a human-machine interface, most of the studies designed the experiment based on the virtual task or assumption task. For example, to evaluate auditory attention in a human-machine system, a choice RT experiment was organized, in which the user must give a response that corresponds to the stimulus [20]. In another research, to make ergonomics recommendations for multisensory interface design in control consoles, a signal (visual or auditory)-press button task was designed to evaluate the human-machine interface under different conditions by measuring RT and error percentages [21]. Gerhardt-Powals [17] created a simple firing task game. RT was obtained by recording the time interval between information receiving and key-pressing. Several principles based on the experiment are concluded to produce a “cognitive friendly” interface.

For the application of the human-machine interface in aviation, the flight deck is sophisticated and contains a lot of information [22]. The problem of human-machine interaction can be viewed as two powerful information processors attempting to communicate with each other via a narrow-bandwidth, highly constrained interface [23]. Numerous experimental results indicate that the bandwidth of human perception is severely limited [24], which means that only limited information can be successfully acquired by users within a unit time. Moreover, the pilot's RT presents more task-related features. Different auditory commands or warning tones in different flight scenes and missions can seriously affect the information requirement of users. For example, in a conditionally automated driving experiment, the group of participants who received commands on limitations had a lower RT when the car approached the deer than the control group [25]. Therefore, it is particularly important to evaluate the human-machine interface in aviation considering different auditory commands in flight scenes as realistic as possible.

The article "Performance Index Based on Predicted Auditory Reaction Time Analysis for the Evaluation of Human-Machine Interface in Flight Control" was published in 2022. Journal: Comput Math Methods Med.

However, in the previous studies, either the experiment was not set under the task state or the experimental measurement of RT may disturb the subjects to complete the original task. Besides, different from other applications, flight tasks and scenarios are too complex to be simulated; for example, in high maneuverability missions, it is hard to generalize the proper voice command in experiments. Also, different from warning/alarm signals, voice commands are informative and too numerous to be traversed simulated. But it is always desired that the proposed method should be able to evaluate the interface design under more generalized situations based on a small-size experimental sample set.

This paper proposed predicted auditory RT as an index to evaluate the console interface of remotely piloted aircraft (RPA). Besides, the methods can be further applied in other domains, such as interface evaluation of airplanes and complex command and control systems. The work focused on the following three problems:

1. The experiment method to measure and evaluate the auditory commands in the task state, which should keep the subject in a normal operating state and not influence the subject to execute the regular task
2. The calculation method to predict the auditory RT of more generalized voice commands with a small-size sample set
3. The analysis method to evaluate and analyze the interface design is based on auditory RT

We try to solve the above problems, and this paper was organized as follows: In Section 2, the architecture of the proposed approach was explained.  Section 3 represents the method of auditory RT measurement, in which the experiment was organized in the pilot's flight task state.  Section 4 was about the prediction method of voice command RT, in which the RT was estimated for more general voice commands based on the key words. Finally, the RT was used to evaluate two flight console interfaces in Section 5, which provided the idea of how to analyze the usability of the interface with RT. In Section 6, conclusions and future work are presented.

## 2. Architecture of Proposed Method

In the human reaction process, a stimulation induces a process in which the stimulus activates the sensory apparatus, which travels through the afferent nerve to the nerve center of the brain, through complex processing, and from the efferent nerve to the muscle, which contracts to perform the operation. Although this process is latent in the body, each step takes time. The sum time is called reaction time. RT consists of perception time (i.e., the time from the presence of the stimulus to the beginning of the action) and action time (i.e., the execution duration of action):

(1) $$\begin{array}{c} \text{RT}=t_{z}+t_{d}, \end{array}$$

where RT is the total reaction time, *t*_*z*_ is the perception time, and *t*_*d*_ is the action time. In terms of information acquisition and processing, perception time refers to the time of auditory information acquisition, while action time refers to the time of active visual information acquisition.

The article "Performance Index Based on Predicted Auditory Reaction Time Analysis for the Evaluation of Human-Machine Interface in Flight Control" was published in 2022. Journal: Comput Math Methods Med.

In a flight task, after the pilot receives a voice command, he/she does not produce the manual operation directly but obtains the related visual information first to gather useful information, then judges the situation based on the information and experience, and finally performs the action. Based on this phenomenon, eye movement tracking is adopted as a measuring means of RT in flight tasks. From the information perception aspect, the time interval between the ending time of voice command and human firstly obtaining the useful visual information indicates the time spent on processing auditory information, while the time interval between gaining first target information and all the useful visual information that have been acquired represents the reaction procedure of the information processing results. As this work uses RT to evaluate the information display interface, the manual operation time is not taken into account.

It is assumed that *t*_1_ and *t*_2_ represent the starting and ending times of a voice command. *t*_3_ is the point-in-time on which the pilot firstly forms the fixation on the Area of Interests (AOIs) of the user interface. Because converting the voice command to useful visual information and achieving this information takes time, *t*_3_ may not always equal to the point-in-time of the first target AOI *t*_4_ for different interfaces. *t*_5_ indicates the time that all target AOIs have been acquired by the pilot. The relationship of these time points in the sequence can be expressed as

(2) $$\begin{array}{c} t_{z}=t_{4}-t_{2},\\ t_{d}=t_{5}-t_{4}. \end{array}$$

A pilot's RT represents the difficulty of obtaining multiple information under a certain command; thus, it can be used as an index to evaluate the rationality of the layout of multiple information in the interface.

The proposed approach mainly consists of three parts. The first part is to obtain the template data of RT for typical auditory commands based on eye movement tracking. The pilot was asked to do the normal flight task in this part, while the typical voice commands were given randomly and eye movement data were recorded at the same time. Since the experiment was done without disturbing the pilot and flight task, all data were gathered in the task state. The second part developed the method of RT prediction based on small samples of experiments, which includes two steps. The first step is key word extraction, which extracts key words from original audio files. This step is constructed based on the fact that experienced pilots usually respond to the voice command according to the acquired key words so that he/she can give the response promptly. The combination of different key words will determine the pilot's RT to the command. The second step is to predict RT, where we trained a neural network that used the template data, which includes RT for typical commands and template key words, to predict RT of more general auditory commands. The significance of this prediction model is that it can estimate the RT for different commands without traversing all sample commands, since not all the flight scenes can be simulated in the simulator, and in some flight missions, the commands should be made according to the real task situation which is hard to be simulated. Moreover, the human-machine interface can be evaluated in more general cases. The workflow of our work is illustrated in Figure 1. The third part is to analyze the flight console interface based on the predicted RT of different voice commands.

The article "Performance Index Based on Predicted Auditory Reaction Time Analysis for the Evaluation of Human-Machine Interface in Flight Control" was published in 2022. Journal: Comput Math Methods Med.

This approach provides a new idea to predict the RT of voice command under the task state for the aviation application. Furthermore, the RT can be adopted as one of the indexes to evaluate the efficiency of a flight console interface, which offers perceptive information to users under various and complex tasks.

## 3. Auditory Reaction Time Obtaining Based on Eye Movement Tracking

In common cases, the interface of upgraded equipment is designed or modified based on the original interface of the previous generation. Assume that interface A is a new interface whose usability needs evaluation. However, since its usability has not been evaluated, we cannot measure it in a real scenario for the sake of safety. At the same time, it takes a lot of manpower and time to conduct experiments on all auditory commands, so we construct a prediction model to predict RT of more voice commands through experiments of a small number of commands which can be simulated. Suppose interface B is an old version interface, which has more pilot's RT data under voice commands. Through the comparison of the pilot's RT under each command, different interfaces can be compared and evaluated. For example, for combat missions, the interface that the pilot has smaller RT with combat commands is better; for search and rescue missions, the interface that the pilot has smaller RT with searching commands is better.

The article "Performance Index Based on Predicted Auditory Reaction Time Analysis for the Evaluation of Human-Machine Interface in Flight Control" was published in 2022. Journal: Comput Math Methods Med.

### 3.1. Experimental Scheme and Platform

The experiments are based on a search and rescue mission. All the experiments were done on the simulator of the RPA operation platform (as shown in Figure 2). The platform is composed of six modules, which are the integrated situation module, flight control module, CCD operation module, radar illumination module, voice command module, and eye movement tracking module. Different flight tasks can be simulated on the platform, such as “take-off,” “climb,” “cruise,” “search target,” and “flight return.” In the experiment, while the RPA pilot executed certain flight tasks, the voice command module broadcasts voice commands according to the current flight situation, which was chosen from the command library including commonly used commands from the ground command center.

The eye movement tracking module recorded the RPA pilot's eye movement data at the same timeline with the voice command and flight parameters with Tobii Pro X3-120. Before the experiment, we used calibration software to calibrate the eye tracker. During the calibration process, we made sure that all the information on the screen was accessible to the pilot. For the collected eye movement data, the fixation time greater than 100 ms was selected as fixation points. In addition, multiple AOIs (Figure 3) can be obtained by dividing functional areas on the display, and eye movement points in corresponding AOI indicate that corresponding AOI information is obtained.

It is discovered that after receiving the auditory command or warning signals, instead of outputting the manual actions immediately, the pilot obtains related visual information firstly to gather useful information to know the current situation or to prepare for the next operation. Then, he finally performs the operation requested by voice command. Based on this discovery, it is reasonable to introduce eye movement tracking to evaluate the pilot's performance of response to the auditory command. Moreover, during the same flight task, to complete the proper operation, for the same command, AOIs (Area of Interests) that expert pilots pay attention to are the same, and these obtained AOIs are quite consistent for the expert pilots. However, different pilots may focus on the same group of AOIs when responding to one command; each pilot may not focus AOIs in the same order. For example, after the pilot got the voice command “encounter storm, altitude 6000,” he/she can first obtain the “altitude” information or the “track” information.

The article "Performance Index Based on Predicted Auditory Reaction Time Analysis for the Evaluation of Human-Machine Interface in Flight Control" was published in 2022. Journal: Comput Math Methods Med.

Therefore, in this work, the auditory RT is defined as the time interval between the end of the voice command and the acquirement of all target AOIs. The target AOIs are obtained through experts' knowledge. For example, after the pilot got the voice command “encounter storm, altitude 6000,” he needs to obtain the “altitude” information and the “track” information. But there is no requirement on the order of information acquisition. In this case, the experiment does not disturb the pilot's operation in flight mission, and the data are recorded in the flight task state.

The subject is an expert pilot, has good flying experience (three years of operating experience), does not wear glasses, and can master the simulation platform proficiently.

After each trial of the experiment, the pilot can have a short break to ensure that the RT is not affected by the fatigue state.

### 3.2. Auditory Reaction Time Obtaining

Through the measurement of action time, the ability of the human-machine interface to display mixed information to pilots is obtained. Performing a command often needs to access several pieces of information on current flight parameters, and this would require the pilot to acquire multiple information either within a single display or from multiple displays. According to SEEV theory [26], the expectation is an important factor affecting visual attention, so the pilot's visual attention should be properly considered and visual information should be input to the pilot in an appropriate way. A good human-machine interface should be reasonably planned; thus, the pilot can quickly get the information with little effort.

We take the flight task “cruise” as an example to illustrate how to gain the RT by eye movement data. The data obtaining process was as follows.

The pilot did a normal flight task in the simulated flight platform; then, he operated the aircraft to the required altitude and started the cruise task. During the cruise phase, the voice commands were sent to the pilot according to the real situation and flight scenes at irregular intervals. The platform can record the time *t*_1*i*_ when voice comment *i* was sent and the ending time *t*_2*i*_ of the command *i*. The pilot's eye movements were recorded with the same time label. The eye movement points were assigned into AOIs as shown in Figure 4, in which the red blocks were the predefined AOIs according to the functional area of the flight console interface, and the green lines indicated the eye movement trajectories from one AOI to the other. In this case, each fixation point was labeled with the functional information. After the end of voice command *i*, the time of the first AOI acquired by the pilot was recorded as *t*_3*i*_, but this firstly obtained information may not be the required information prepared for the operation of commands. Thus, the time of the first target AOI acquired by the pilot was recorded as *t*_4*i*_. When all the target AOIs had been gained by the pilot, the time was recorded as *t*_5*i*_. The total RT of command *i* can be calculated by RT_*i*_ = *t*_5*i*_ − *t*_4i_.

The article "Performance Index Based on Predicted Auditory Reaction Time Analysis for the Evaluation of Human-Machine Interface in Flight Control" was published in 2022. Journal: Comput Math Methods Med.

## 4. Reaction Time Prediction

### 4.1. Extraction of Key Words in Voice Command

In the flight mission, when the voice command is given by the command center or ground station, the expert pilot usually responds to the obtained key words involved in command based on his experience. In this case, he can execute the command as soon as possible to handle the complex situation. For example, when there was command “no. 02 CCD on the target for 10 seconds,” where “02” is the code number of his airplane, the pilot would pay his attention to the information of CCD view in the user interface according to the key word “CCD.”

In the flight mission, because the voice commands given by the command center has very strict restrictions and is commonly broadcast with certain frequency and tones, the features of the same key words in different commands are quite similar. Moreover, it is possible to collect the key words appearing in the voice command file based on the experiences of the expert pilot. Thus, the template base can be constructed to gather the extracted features of key words. Since the amount of information contained in different key words is different, which determines the difficulty level of information processing for the pilot, a thesaurus is established according to the word information content, which is also provided by the expert pilots. Then, the detected key words are classified according to the kind of thesaurus. In this case, the template base is stored according to the information category.

For any voice command during the flight task, the sliding window method and dynamic time warping (DTW) matching algorithm are adopted to automatically detect the input key words. The recognition method of voice command designed in this paper is illustrated in Figure 5. Besides the preprocessing of input voice command, the process mainly includes feature extraction of key words and template matching, which will be explained in the following parts.

#### 4.1.1. Feature Extraction of Key Words in Voice Command

Before establishing the template base and recognizing the input speech, it is necessary to preprocess the speech signal to facilitate further processing, which commonly includes the processing procedure, such as sampling and quantization, preemphasis, framing, and windowing. The two most commonly used characteristic parameters are MFCC (Mel Frequency Cepstral Coefficient) and LPCC (cepstral linear predictive coding). Among them, MFCC is a feature parameter widely used in speech recognition. The extraction process of MFCC feature parameters [27] for key words in voice command adopted in this paper is described as the following steps:

1. The preprocessing adopted in this work contains the procedure of preemphasis, framing, and windowing. The preemphasis filter is applied to a signal *x* using the first-order filter in the following equation with the filter coefficient *α*:

(3) $$\begin{array}{c} x_{1}\left(t\right)=x_{0}\left(t\right)-\alpha x_{0}\left(t-1\right). \end{array}$$

After preemphasis, the signal is split into short time frames *x*_2_(*n*). Then, the Hamming window is applied to each frame aimed at increasing the continuity of the left and right ends of the frame. The chosen form is

(4) $$\begin{array}{c} w\left(n\right)=0.54-0.46\cos\left(\frac{2\pi n}{N-1}\right), \end{array}$$

(5) $$\begin{array}{c} x\left(n\right)=x_{2}\left(n\right)w\left(n\right), \end{array}$$

where *N* is the window length, 0 ≤ *n* ≤ *N*.

(2) The power spectrum of the voice command signal is calculated by Fourier transform:

(6) $$\begin{array}{c} P=\frac{{\left|FFT\left(x_{i}\right)\right|}^{2}}{N}, \end{array}$$

where *x*_*i*_ is the *i*^th^ frame of *x*.

(3) Then, we can convert between Hertz (*f*) and Mel (*M*(*f*)) using the following equations:

(7) $$\begin{array}{c} M\left(f\right)=2595\log_{10}\left(1+\frac{f}{700}\right), \end{array}$$

in which 2959 and 700 are empirical constants. The Mel scale is aimed at mimicking the nonlinear human ear perception of sound, by being more discriminative at lower frequencies and less discriminative at higher frequencies.

The article "Performance Index Based on Predicted Auditory Reaction Time Analysis for the Evaluation of Human-Machine Interface in Flight Control" was published in 2022. Journal: Comput Math Methods Med.

The energy spectrum is passed through a set of Mel scale triangular filter banks, and a filter bank with *M* filters is defined as

(8) $$\begin{array}{c} H_{m}\left(k\right)=\left\{\begin{array}{cc} 0, & k<f\left(m-1\right),\\ \frac{2\left(k-f\left(m-1\right)\right)}{\left(f\left(m+1\right)-f\left(m-1\right)\right)\left(f\left(m\right)-f\left(m-1\right)\right)}, & f\left(m-1\right)\leq k\leq f\left(m\right),\\ \frac{2\left(f\left(m+1\right)-k\right)}{\left(f\left(m+1\right)-f\left(m-1\right)\right)\left(f\left(m\right)-f\left(m-1\right)\right)}, & f\left(m\right)\leq k\leq f\left(m+1\right),\\ 0, & k\geq f\left(m+1\right), \end{array}\right. \end{array}$$

where ∑_*m*=0_^*M*−1^‍*H*_*m*_(*k*) = 1.

(4) At last, we have to obtain the Mel Frequency Cepstral Coefficients (MFCCs). The logarithmic energy output of each filter bank is calculated by the following equations:

(9) $$\begin{array}{c} s\left(m\right)=\ln\left(\overset{N-1}{\underset{k=0}{\sum }}‍{\left|X\left(k\right)\right|}^{2}H_{m}\left(k\right)\right),\;0\leq m\leq M. \end{array}$$

Discrete Cosine Transform (DCT) is applied to decorrelate the filter bank coefficients and yields a compressed representation of the filter banks:

(10) $$\begin{array}{c} C\left(n\right)=\overset{N-1}{\underset{m=0}{\sum }}‍s\left(m\right)\cos\left(\frac{\pi n\left(m-0.5\right)}{M}\right),\;n=1,2,\cdots ,L, \end{array}$$

where *L* refers to the order of the MFCC coefficient.

#### 4.1.2. Key Word Template Matching

When using the template matching method for speech recognition, a single word is generally regarded as a recognition unit. In the training phase, the user said every word in turn, and each word's feature vector is extracted as a template in the template base. In the recognition phase, the similarity between the input speech feature vector series and each template in the template base is measured. The template owing the highest similarity is picked as recognition results.

However, it is impossible to simply compare the input parameter sequence with the corresponding reference template directly, because the speech signal has considerable randomness; even if the same person speaks the same word at different times and makes the same sound, it cannot have the same length of time. In template matching, these changes of time length will affect the measurement estimation and reduce the recognition rate. Therefore, the procedure of time scaling for the voice command signal is essential.

DTW is a nonlinear regularization technique which combines time regularization with distance measure calculation. For example, the test audio parameters are *I*-frame vector, and the reference template is a *J*-frame vector, *I* ≠ *J*; then, dynamic time warping is to find a time warping function *j* = *ω*(*i*), which maps the time axis *i* of the test vector nonlinearly to the time axis *j* of the template and makes the function *ω* meet:

(11) $$\begin{array}{c} D=\underset{\omega \left(t\right)}{\min}\overset{I}{\underset{i=1}{\sum }}‍d\left[T\left(i\right),\;R\left(\omega \left(i\right)\right)\right], \end{array}$$

where *d*[*T*(*i*),  *R*(*ω*(*i*))] is the distance measurement between the *i*^th^ test vector *T*(*i*) and the *j*^th^ vector *R*(*j*). *D* is in the optimal time warping case. The cost function is

(12) $$\begin{array}{c} D\left[c\left(k\right)\right]=d\left[c\left(k\right)\right]+\min D\left[c\left(k-1\right)\right], \end{array}$$

where *d*[*c*(*k*)] is the cost of *c*(*k*). Thus, the total cost function is the sum of the cost of the point itself and the cost of the best path to that point.

The article "Performance Index Based on Predicted Auditory Reaction Time Analysis for the Evaluation of Human-Machine Interface in Flight Control" was published in 2022. Journal: Comput Math Methods Med.

Because DTW continuously calculates the distance between the two vectors to find the optimal matching path, two-vector matching is the normalized function with the minimum cumulative distance, which ensures the maximum acoustic similarity between them.

### 4.2. Key Word(s) Vectorization

When a pilot performs a task, his responding time to the voice command is actually determined by the combination of multiple key words in the command. He will pay attention to different combinations of key words to complete the flight target task.

According to the command template, the identified flight commands are converted into the input sample of the prediction model. The specific method is described as follows.

As it is difficult to determine the RT directly from the text information, it is necessary to preprocess the obtained text information. Inspired by the model of natural language processing, we extract key words from the possible appearing voice commands according to the experience of expert pilots. These words are divided into different topics based on the content similarity, and each topic is defined as one of the dimensions in the feature vector. Thus, the feature vectors corresponding to the commands are obtained. Then, topic words are selected according to the probability; that is, if a sentence appeared, several words that represent the sentence are selected as the topic words. For example, when the word “climb to 1000” is detected, there is a high probability that the sentence belongs to the category of “climb to XX,” while the word “to” is detected, there is not a high probability that the command relates to the category of “climb to XX.” Therefore, for this sentence, the topic word “climb” is chosen to represent the topic of the command, and this word covers most of the information of this sentence. Key words with high correlation, that is, words with a high probability of appearing together, words that are similar, or words that can be replaced with each other, are classified as one topic. Topic words are determined according to experimental results. Since the structure of voice command in flight scenes is specified and the command words are very standard, the voice command can be vectorized through these topic words. Here are some topic words used in the experiment presented in Table 1. For the real scene, there will be more topic words.

For example, if the above topic words appear in the voice command, the vector of the corresponding dimension is assigned as 1. If it does not appear, it is assigned as 0. Each command is vectorized according to the selected topic words.

The article "Performance Index Based on Predicted Auditory Reaction Time Analysis for the Evaluation of Human-Machine Interface in Flight Control" was published in 2022. Journal: Comput Math Methods Med.

Some typical command vectors are presented in Table 2.

### 4.3. Reaction Time Prediction

So far, the problem of RT prediction can be regarded as a common prediction problem. That is, the command vector of each voice command is given to estimate the corresponding response time. Supervised learning algorithms can be used to solve this problem.

A BP neural network is constructed in this paper to achieve the prediction of RT. The neural network structure is shown in Figure 6. The input data is the vectorized voice command, and the output data is the RT. All the data obtained from the experiment are used to train the neural network.

### 4.4. RT Prediction Results and Analysis

In this paper, we gave an example of 14 voice commands used to train the neural network to predict the RT. Prediction results are depicted in Figure 7. The boxes represent the measured RT data obtained from all the experiments. The yellow line represents the median value of all the experimental data, and the blue dots are the predictive value of the neural network for the commands.

Calculate accuracy *δ*_*i*_ for command *i* in cross-checking:

(13) $$\begin{array}{c} \delta_{i}=\frac{r_{pi}-\overset{¯}{r_{ei}}}{\overset{¯}{r_{ei}}}. \end{array}$$

Total accuracy *δ* is computed as

(14) $$\begin{array}{c} \delta =\frac{\Sigma_{i=1}^{n}}{n}, \end{array}$$

where *r*_*pi*_ represents the predicted RT for command *i* and $\overset{¯}{r_{e}}$ is the mean value of obtained RT for command *i*, while *n* represents the total number of commands.

In this example, the overall result has the prediction accuracy (*δ* = 0.904), shown in Figure 7. For some commands, the prediction accuracy can hit up to 0.995. However, some only achieved 0.470. The reason can be explained by Figure 8. In the figure, the blue bars represent the number of times that those topic words are trained in the condition of the combination topic words that appeared in the voice command, while the orange bars represent the number of times that those topic words are trained individually. For example, in command “hover at navigation point,” “hover” and “navigation” belong to a different topic category and were trained together. In command “climb up to 1100,” “up” was trained independently, e.g., the command “contact target within 10 seconds” has a bad prediction performance (0.470), because the topic words in this command have not been individually trained. The command “climb up to 1100” performs well (0.995), because the topic word “up” is trained individually, which can achieve good prediction accuracy for the combination of words as well. In this example, topic words no. 11 and no. 12 do not appear in all 14 instructions, as shown in Table 2. However, in order to illustrate that our method can predict the reaction time of larger samples of instructions based on training more topic words, we keep these two topic words in Figure 8.

The article "Performance Index Based on Predicted Auditory Reaction Time Analysis for the Evaluation of Human-Machine Interface in Flight Control" was published in 2022. Journal: Comput Math Methods Med.

## 5. Interface Evaluation Based on Reaction Time Prediction

In this section, two flight console interfaces are evaluated based on the predicted voice command RT. Interface B is the original version of the RPA operation interface, while interface A is the updated version. The differences between the two versions are listed below:

1. Interface A (Figure 4(a)) displayed speed and altitude information of RPA using the overlapping display on the front-view scene interface. For example, “speed” is shown in Rec 6 and “altitude” is shown in Rec 7. Rec indicates the previously defined AOI and is presented as a red rectangle in the figure. Yellow dots are recorded pilots' eye fixations during the flight task
2. Interface B (Figure 4(b)) displayed speed and altitude information separately. For example, “speed” and “altitude” are depicted in Rec 14 and Rec 15, respectively, and they were shown independently on the flight parameter monitoring interface

Except for the “altitude” and “speed” information, other information on these two interfaces remains the same.

The operation platform is placed in a quiet and well-lit experimental environment; the expert pilot has good flying experience (three years of operating experience), does not wear glasses, and can master the simulation platform proficiently. Large head rotation during the execution of flying tasks is avoided to ensure the accuracy of eye tracker data.

With interface A, the pilot's RT experiments were conducted on 14 groups of voice commands, 8 times for each command. The total number of valid training RT data is 86. With interface B, the pilot's RT experiments were executed on the same 14 groups of commands, but 4 times for each command. After removing the measured RTs that are larger than 5 s as well as RT with a very large fluctuation range, which is generally caused by the accuracy of the eye tracker, the RT data from the experiment was obtained.  Figure 9 presents all measured RT of each voice command for the two interfaces, respectively, in which the box depicts the measured RT data distribution, the orange line represents the median value for all the trials, and the dotted green line represents the mean value.

For both of the two cases, voice commands with nos. 1-8, 10, 11, 13, and 14 are training datasets, while nos. 9 and 12 are test sets (Table 2). RTs of voice command nos. 9 and 12 were predicted with the proposed model. The predicted error rate is 5.5% and 15.9% for instructions no. 9 and no.12, respectively, which refers to the mean value of RT of all trials. From the RT predicted results present in Figure 10, we can discover that for most instructions, the RTs of two interfaces are quite close. Distinctively, for instructions 4, 5, and 14, interface B performed better than interface A. For instructions 6 and 7, interface A performs better than interface B.

The article "Performance Index Based on Predicted Auditory Reaction Time Analysis for the Evaluation of Human-Machine Interface in Flight Control" was published in 2022. Journal: Comput Math Methods Med.

In Table 3, bold indicates that interface A or B performed better in this voice instruction. “f” represents that pilots obtained the visual information “front view,” “a” represents “altitude,” “s” is “speed,” “t” is “track,” “l” represents “CCD information,” and “()” is this AOI appearing several times. It reveals that with interface B, pilots spend much time on “CCD information” (for example, instructions no. 6 and no. 7). The reason is that when the pilot needed CCD information to respond to the voice command, in interface A, the pilot uses his peripheral to roughly obtain the CCD information because the speed and altitude information is very close to the CCD view (CCD view is presented on the left interface in Figure 4). This can also be discovered by the fact that there are more fixation points formed on the CCD view of interface B compared with interface A. However, in interface B, these pieces of information are separated, which indicates that the pilot has to look at the CCD information intentionally to obtain it.

For voice command no. 4, the AOIs required by the pilot are the same in the two interfaces, while interface B shows better performance. In our case, this indicates that the speed and altitude information in interface B (displayed as overlay mode) can be much easier obtained by the pilot than interface A (displayed as digital numbers).

As the CCD information can be easier obtained by pilots with interface A, information display as interface A can be used in search and rescue missions. Because the altitude and speed information are relatively easier to be acquired with interface B, information presented like interface B can be used in high maneuverability missions.

## 6. Conclusions and Future Work

This paper proposed predicted auditory RT as an index to evaluate the flight console interface. The proposed architecture of the approach consisted of three parts RT measurement under samples of voice commands, prediction method to estimate RT under more general commands, and interface evaluation with RT prediction, which obtained the following achievement.

Firstly, the pilot's auditory RT is effectively calculated by eye movement tracking, which makes the experiment carried out in a flight task state, and the measurement would not influence the pilot to execute the normal task.

The article "Performance Index Based on Predicted Auditory Reaction Time Analysis for the Evaluation of Human-Machine Interface in Flight Control" was published in 2022. Journal: Comput Math Methods Med.

Secondly, the RT prediction model is built based on the extracted key words that appeared in commands. Then, a neural network is constructed, which made the RT under more generalized commands be estimated with small sample experiments. This can help to overcome the dilemma that some flight scenes are hard to be simulated and various voice commands are impossible to be traversed simulated.

Finally, the voice command RT is adopted as one aspect to evaluate the utilization of the new generation interface, which considers not only the time accumulation effect of the human state during the interaction but also instantaneous reactions to the input information of the interface.

This paper only presented the application in the evaluation of the flight console interface; in fact, the proposed approach can also be applied in other systems, such as the human-robot interface and operation interface of the command center. For further applications, there are still several works that need to be done in the future:

1. The voice command library used in this paper is not large enough, a bigger dataset can be used to improve the prediction results, and more evaluation indexes could be used to evaluate the human-machine interface
2. The features of instructions are not only included key words but semantic structure. The relationship between each key word can be considered, which may help to increase the RT prediction accuracy in a more general scenario
3. The experiments were done under specific tasks, but our work actually can resolve the prediction problem under several different tasks. Thus, context information can be input into the prediction model to achieve the prediction under different tasks
4. The target AOI base is based on experts' knowledge. However, while new technology emerges, new instructions will emerge, which means no target AOI knowledge to those instructions. Thus, an experimental method can be proposed to extract experts' knowledge

## Figures and Tables

**Figure 1:** Architecture of the proposed method.

**Figure 2:** Flight mission simulation and reaction time measurement platform.

**Figure 3:** Eye movement trajectory responded to the voice command in flight task.

**Figure 4:** Flight console interface with eye movement: (a) interface A (new version); (b) interface B (old version).

**Figure 5:** Proposed recognition method of key words in voice command.

**Figure 6:** Structure of reaction time prediction model based on BP neural network.

The article "Performance Index Based on Predicted Auditory Reaction Time Analysis for the Evaluation of Human-Machine Interface in Flight Control" was published in 2022. Journal: Comput Math Methods Med.

**Figure 7:** Reaction time prediction results for different voice instructions.

**Figure 8:** Training number of topic words appeared together or independently.

**Figure 9:** Results of pilot's reaction time experiments on interfaces A and B.

**Figure 10:** Reaction time comparison.

**Table 1:** Topic words.

Topic no.	1	2	3	4	5	6	7
Key word	CCD	Hover	Search target	Fast feed	Back	Direction	Climb (up) down
Topic no.	8	9	10	11	12	13	14
Key word	Attitude	Navigate	Right left	Team	Unknown	Quit	Time second

**Table 2:** Topic word vectors of 14 typical commands.

No.	Command	Topic word vector
1	No. 02 hover at navigation point	[0, 1, 0, 0, 0, 0, 0, 0, 1, 0, 0, 0, 0, 0]
2	Fast turn up	[0, 0, 0, 1, 0, 0, 1, 0, 0, 0, 0, 0, 0, 0]
3	All planes quit the mission and fly to the nearest airfield	[0, 0, 0, 0, 0, 0, 0, 0, 0, 0, 0, 0, 1, 0]
4	Fast turn down	[0, 0, 0, 1, 0, 0, 1, 0, 0, 0, 0, 0, 0, 0]
5	No. 01 11 o'clock direction target appears	[0, 0, 1, 0, 0, 1, 0, 0, 0, 0, 0, 0, 0, 0]
6	Fast turn left	[0, 0, 0, 1, 0, 0, 0, 0, 0, 1, 0, 0, 0, 0]
7	Fast turn right	[0, 0, 0, 1, 0, 0, 0, 0, 0, 1, 0, 0, 0, 0]
8	11 o'clock direction search targets	[0, 0, 1, 0, 0, 1, 0, 0, 0, 0, 0, 0, 0, 0]
9	Climb up to 1100	[0, 0, 0, 0, 0, 0, 1, 0, 0, 0, 0, 0, 0, 0]
10	Go back ten miles and return	[0, 0, 0, 0, 1, 0, 0, 0, 0, 0, 0, 0, 0, 0]
11	No. 02 CCD on the target for 10 seconds	[1, 0, 1, 0, 0, 0, 0, 0, 0, 0, 0, 0, 0, 1]
12	To landing altitude	[0, 0, 0, 0, 0, 0, 0, 1, 0, 0, 0, 0, 0, 0]
13	Contact target within 10 seconds	[0, 0, 1, 0, 0, 0, 0, 0, 0, 0, 0, 0, 0, 1]
14	Climb up to 1300, attention on fuel pressure	[0, 0, 0, 0, 0, 0, 1, 0, 0, 0, 0, 0, 0, 0]

**Table 3:** AOIs for instructions.

Instruction	Interface A	Interface B	Comparison
4	f a s (t)	**f a s (t)**	Same
5	f t l	**f l**	A has t
6	**f t (a)**	f l t (a)	B has l
7	**f t**	f l t	B has l
14	f a (s)	**f a**	A has (s)

## Data Availability

The data that support the findings of this study are available on request from the corresponding authors. The data are not publicly available due to privacy restrictions.
